# The OMICs Window into Nonalcoholic Fatty Liver Disease (NAFLD)

This article has been retracted.

**DOI:** 10.3390/metabo9020025

**Published:** 2019-02-01

**Authors:** Lucia Carulli, Giulia Zanca, Filippo Schepis, Erica Villa

**Affiliations:** Division of Gastroenterology, Department of Medical Specialties, University of Modena and Reggio Emilia, 41124 Modena, Italy; lucia.carulli@unimore.it (L.C.); 165382@studenti.unimore.it (G.Z.); filippo.schepis@unimore.it (F.S.)

**Keywords:** nonalcoholic fatty liver disease, nonalcoholic steatohepatitis, fibrosis, liver biopsy, genomics, metabolomics, proteomics, transcriptomics

## Abstract

Nonalcoholic fatty liver disease (NAFLD) is a common cause of hepatic abnormalities worldwide. Nonalcoholic steatohepatitis (NASH) is part of the spectrum of NAFLD and leads to progressive liver disease, such as cirrhosis and hepatocellular carcinoma. In NASH patient, fibrosis represents the major predictor of liver-related mortality; therefore, it is important to have an early and accurate diagnosis of NASH. The current gold standard for the diagnosis of NASH is still liver biopsy. The development of biomarkers able to predict disease severity, prognosis, as well as response to therapy without the need for a biopsy is the focus of most up-to-date genomic, transcriptomic, proteomic, and metabolomic research. In the future, patients might be diagnosed and treated according to their molecular signatures. In this short review, we discuss how information from genomics, proteomics, and metabolomics contribute to the understanding of NAFLD pathogenesis.

## 1. Introduction

Nonalcoholic fatty liver disease (NAFLD) is becoming the most common chronic liver disorder affecting adults and children in the western countries. Its prevalence has reached very high levels (6–35%) worldwide. In Europe, the median prevalence is 25–26% with slight differences in different populations [1]. NAFLD is subdivided into nonalcoholic fatty liver (NAFL), or simple steatosis without evidence of inflammation, and non-alcoholic steatohepatitis (NASH), characterized by hepatic steatosis, cell injury with a mixed inflammatory lobular infiltrate and variable fibrosis [2,3]. The differential diagnosis between disease stages (NAFL and NASH) is commonly based on liver biopsy [4]. Liver biopsy, however, can be potentially biased as the small portion of hepatic tissue obtained could underrepresent the hepatic condition. Liver biopsy also has some potential complications, such as bleeding, abdominal discomfort, or pain. Noninvasive approaches, therefore, have gained considerable attention, and current research efforts are addressed to find reliable biomarkers able to predict disease severity and prognosis. The recent advances in the field of genomics, transcriptomics, proteomics, and metabolomics have greatly facilitated this approach [5]. This review is aimed to unveil how knowledge derived from a large-scale genetic profiling of NAFLD genomics, as well as transcriptomics and metabolomics of NAFLD, may contribute to the diagnosis and risk prediction of NAFLD progression (Figure 1). We will review the main applications of OMICs signatures in clinical practice for the assessment of disease risk, disease severity and prognosis, and for monitoring treatment response.

## 2. Genomics 

### 2.1. Genome Variation 

The pathogenesis of NAFLD is not fully understood, although it is known that it depends on the combination of many factors, including genetic and environmental factors. The relevant polymorphism of the rs738409 C/G of the patatin-like phospholipase domain containing 3 (PNPLA3) was identified by means of a genome wide association study [6]. Following this study, the involvement of genetic determinants of NAFLD were replicated by several studies, which confirmed that the G allele is significantly associated not only with an increased risk of fatty liver but with histological disease severity as well. Sokooian et al. [7], in a meta-analysis on the influence of I148M variant on NAFLD susceptibility and histological severity, showed that rs738409 not only explains about 5.3% of the total variance in NAFLD, but it is also associated with more aggressive disease. According to data derived from the first exome-wide association study of liver fat content, another variant has been implicated in increased liver fat content. This variant is the rs58542926 (E167K), a non-synonymous variant located in TM6SF2 (Transmembrane 6 Superfamily Member 2), which seems significantly associated with increased liver fat content [8]. The rs58542926 has a significant role in modulating lipid traits, which is however opposite between genotypes. Carriers of the minor T allele are protected from cardiovascular disease, although it confers risk for NAFLD [9,10].

The use of genetic markers for risk assessment—either alone or as a part of multi-score biomarkers—is justified by published data. Particularly, the 738409-G risk allele could be used for individual risk assessment. Kotronen et al. [11] combined genetic (rs738409 genotypes), clinical and laboratory data in order to evaluate the AFLD risk. Their score model was able to envisage increased liver fat content with a sensitivity of 86% and a specificity of 71%; however, they realized that adding the genetic information improved the accuracy of NAFLD prediction by less than 1% [11]. There have been several other attempts to incorporate genetic markers into noninvasive tests to discriminate between NAFLD and NASH. Nobili and coworkers [12] recently attempted to set up a risk score including 4-polymorphisms (PNPLA3, SOD2, KLF6, and LPIN1) and clinical risk factors, obtaining an Area Under the Receiver Operating Characteristic (AUROC) of 0.80 in predicting NASH in obese children [12]. Two other scores include the NASH Clin Score obtained by the combination of aspartate aminotransferase (AST) and fasting insulin plus genetic data (rs738409 genotypes) [13], and the NASH ClinLipMet Score that is the NASH Clin Score with the addition of circulating metabolites such as glutamate, isoleucine, glycine, lysophosphatidylcholine, and phosphoethanolamine [13]. Genetic markers have also shown promising results in the prediction of response to therapeutic intervention. An example is the variation in PNPLA3 that identifies obese subjects with increased sensitivity to decrease of liver fat content during weight loss. In the study by Sevastianova et al. [14], subjects homozygous for the rs738409-G allele experienced a greater reduction in liver fat following weight loss. A greater reduction in liver steatosis was also observed in rs738409-G allele carriers, after bariatric surgery [15].

### 2.2. Epigenetic Modifications

Epigenetic modifications are attractive targets for therapeutic intervention. DNA methylation can be modified by transcription as well as environmental factors. The importance of this modification has been shown in patients after a massive weight loss following bariatric surgery. Ahrens and coworkers observed an epigenetic remodeling of liver tissue in a cohort of obese patients with NAFLD undergoing bariatric surgery [16]. Also, changes in DNA methylation could be used as a biomarker that allows, for instance, to monitor the effectiveness of pharmacotherapy or lifestyle changes. Changes in DNA methylation can be found not only in the nuclear genome, but also in mitochondrial genomes [17,18]. The role of mitochondria and mitochondrial DNA (mtDNA) in metabolic-syndrome related phenotypes has been known for a long time. The evidence strongly suggests that mitochondrial dysfunction might be also involved in the pathogenesis of NAFLD progression. Pirola and coworkers [18] observed that hepatic methylation and transcriptional activity of the MT-ND6 (mt genome encoded NADH dehydrogenase 6, a member of the OXPHOS complex 1) are associated with the histological severity of NAFLD. Even more interestingly, the epigenetic changes of mtDNA are potentially reversible by lifestyle changes, such as physical activity.

## 3. Transcriptomics

### Cell-Free DNA and RNA

Cell-free DNA (cfDNA) and cell-free RNA (cfNAs) are nucleic acids molecules that circulate freely in the bloodstream. They derive primarily from dying cells of distant tissues. They are currently the focus of intensive research for circulating molecular biomarkers. Several studies have evaluated plasma cell-free DNA methylation as a liquid biomarker of hepatic fibrosis in non-alcoholic fatty liver disease. Preliminary results, however, indicate a substantial lack of specificity, as they can be completely unrelated to NASH biology. Hardy et al. [19] evaluated if methylation of human plasma DNA was able to discriminate liver fibrosis severity in NAFLD subjects. PPARγ DNA methylation was quantified and stratified patients into mild and severe fibrosis, Kleiner 1–2 and Kleiner 3–4, respectively. Increased methylation of PPARγ promoter plasma DNA was paralleled by increased hepatocellular DNA methylation. Same data were obtained in patients affected by alcoholic liver disease (ALD). Similar results were demonstrated in patients with ALD cirrhosis. Hypermethylation at the PPARγ gene promoter is a marker for fibrotic progression of chronic liver disease independently of the etiologies (viral, alcoholic, and metabolic), and is specific of liver fibrosis. The ability to detect and quantify hypermethylation at the promoter of the PPARγ in cfDNA as a new liquid biomarker offers the potential for a cost-effective blood-based liquid biomarker of liver fibrosis [20]. Important technical problems, due to its very low concentrations and the high fragmentation, might represent important limitations and may be difficult to overcome [21]. MicroRNAs (miRNAs) are highly conserved noncoding small RNAs, involved in the post-transcriptional process of gene regulation. In addition, unlike cfDNA, cfmiRNAs are resistant to degradation, making them ideal biomarkers for use in the clinical setting. Circulating miRNAs have been proposed as new non-invasive diagnostic tools to distinguish control subjects vs. patients and NAFLD vs. NASH. Several studies have explored, in case-control studies, the circulating miRNA signature of NAFLD, and data are encouraging for using them as predictors of NAFLD-disease stages [22,23,24,25]. Particularly, as observed by Pirola et al. [22], circulating miR122 and miR192 not only mirror histological and molecular events occurring in the liver, but also have a reliable predictive power in differentiating simple steatosis from NASH. They demonstrated that among 84 circulating miRNAs analyzed, miR-122, miR-192, and miR-375 were significantly upregulated in the serum in nonalcoholic steatohepatitis (NASH) compared to simple steatosis (SS). Liver miR-122 liver expression was downregulated tenfold in NASH compared with SS. Moreover miR122, in Huh 7cells, regulates alanine aminotransferase (ALT) levels by interacting with GPT1 at the coding region, enhancing its translation. According to a pilot study by Tan Y et al. [23], a panel of circulating microRNAs might be used as potential biomarkers for the diagnosis of nonalcoholic fatty liver disease. Investigating miRNA expression in NAFLD patients and controls, they identified a miRNA panel (miR122-5p, miR1290, miR27b-3p, and miR192-5p) with a high diagnostic accuracy for NAFLD [23]. Moreover, the miRNA panel showed to be a more sensitive and specific biomarkers for NAFLD, compared to ALT and Fib-4. Similar results were obtained by other authors [24], that evaluated miRNAs in chronic hepatitis C(CHC) and NAFLD. As for chronic hepatitis C patients, it was observed that in NAFLD subjects, serum levels of miR-122, miR-34a, and miR-16 were significantly increased compared to control subjects and that miR-122 and miR-34a levels had a positive correlation with disease severity, liver enzymes levels, fibrosis stage, and inflammation activity in both CHC and NAFLD subjects. miR-34a and miR-122 may represent novel, noninvasive biomarkers of diagnosis and histological disease severity in patients with CHC or NAFLD. Another combination score, including miR122, miR192, miR21, ALT, and CK-18-Asp396, was evaluated in NAFLD patients and healthy controls. It also evaluated its correlation with known biomarkers like ALT and CK-18-Asp396. This combined score seems to have a higher potential of NASH prediction, exhibiting an AUROC of 0.83 for the prediction of NASH [25]. On the whole, cfmiRNAs seem to be reliable candidates for the incorporation into multi-panel scores for the prediction of NAFLD and NASH.

## 4. Proteomics

The use of plasma or serum proteins for predicting liver fibrosis has been abandoned, because it is technically difficult and has a low performance and poor accuracy. Recently, attempts to develop combined tests that integrate clinical and laboratory data, including circulating proteins, were also made. Sookoian et al. [26] proposed a test, based on clinical, laboratory data and routine biochemical tests, C-reactive protein, soluble intercellular adhesion molecule-1 (sICAM-1), and anthropometric evaluation, that was able to discriminate between simple steatosis and steatohepatitis with a probability for NASH of 99.5% if all test were positive. For the prediction of NAFLD, but not NASH, Wood et al. [27] developed a multi-component classifier for hepatic steatosis. It is a test that includes genetic (rs738409) and clinical data, and different proteins (ACY1, SHBG, CTSZ, MET, GNS, LGALS3BP, CHL1, SERPINC1). The AUROC for steatosis was 0.935, a value shown to be quite reliable in disease risk evaluation. For screening programs, this approach has limited cost-effectiveness. Fibrogenesis in the liver plays an important role in the progression to NASH.

Decaris et al. [28], in order to identify subjects with rapidly progressing disease and with an early response to therapy, developed a novel method able to quantify fibrogenesis flux rates both in liver tissue and blood. NAFLD subjects were fed heavy water (2H2O, 50-mL aliquots) right before a liver biopsy. Liver collagen fractional synthesis rate (FSR) and plasma lumican FSR were measured with mass spectrometry. In NAFLD patients, hepatic collagen FSR increased with progressing disease stage. Plasma lumican FSR showed a significant positive correlation with hepatic collagen FSR. These data indicate that they may be used as direct or surrogate markers of liver disease progression. Okanoue et al. [29], combining type IV collagen 7S and aspartate aminotransferase (AST) in a scoring system named CA, were able to predict both NASH and related fibrosis with sufficient accuracy. The scoring system needs to be validated in independent larger populations from multiple clinical centers. Finally, also measuring circulating procollagen III (PIIINP) was shown to be quite accurate in the prediction of NASH vs NASH-fibrosis. PIIINP is able to discriminate between simple steatosis and NASH or advanced fibrosis [30]. Proteomic studies are not yet so developed in NAFLD. Rodriguez-Suarez et al. [31] showed that in NAFLD and healthy subjects, protein expression was different. Using differential in-gel electrophoresis (DIGE) combined with MALDI TOF/TOF and Western blot analysis of tissue and serum samples, they identified candidate markers associated with NAFLD. The two interesting protein candidates are the mitochondrial enzyme CPS1 (Carbonyl-Phosphate Synthase 1) and GRP78, also known as heat shock protein family A (Hsp70) member 5, which could stratify the different phenotypes associated with disease severity [31]. Similar results were obtained by Younossi et al. [32] using a similar approach, including SELDI-TOF mass spectrometry. Results revealed twelve significantly different protein peaks, with differential expression of several genes and protein peaks in patients within and across the forms of NAFLD. The identified peaks need replication and large-scale testing.

## 5. Metabolomics

Many years ago, Puri et al. [33] conducted extensive studies on plasma metabolomics in NAFLD. They analyzed plasma lipids and eicosanoid metabolites by mass spectrometry. They showed increased levels of 11-HETE, a non-enzymatic oxidation product of arachidonic (20:4) acid, in NASH compared to NAFL subjects. In severe NAFLD, metabolomic analysis also showed marked changes in bile salts (BA) and glutathione-related metabolites, as well as higher levels glucose, mannose, lactate, and pyruvate. Recent studies on bile salts indicated that conjugated primary bile acids were significantly higher in NASH [34,35]. Han et al. [36] analyzed the progression of NASH in a translational human–animal study. They found that metabolome changes mainly concerned amino acid and BA metabolism with significant differences between animals and humans. In fact, Taurine acid has been shown to be increased in human but not in the rat NASH models. Recently, Dong et al. [37], analyzing urine and blood of non-diabetic NAFLD with normal liver function tests, NASH and HC subjects with impairment of liver function, identified biomarkers, whose presence was different according the NAFLD stage. They showed by ROC analysis that 3-indoleacetic acid, L-carnitine, pyroglutamic acid, and indolelactic acid might discriminate NASH from NAFLD.

Lake et al. [38] also studied the progression of SS toward NASH by metabolomics and transcriptomic analysis and reported increased levels of leucine (+127%), isoleucine (+139%), and valine (+147%) from NAFL to NASH. Similarly, carnitine metabolites were significantly elevated in NASH compared to NAFL. In a recent study Alonso et al. [39], after combining metabolomic data obtained experimental animals as well as human samples, stated that there are two subtypes of NASH according to their circulating pattern of triglycerides, diglycerides, fatty acids, ceramides, and oxidized fatty acids. These might be used to monitor disease progression and identify therapeutic targets for patient. Recent explorations on liver metabolism during NASH development, have shed new light on the meaning of elevated ALT and AST that may be consequence of impaired amino acids metabolism in the liver rather than liver injury [40,41,42].

Interestingly, alterations of amino acids and lipid metabolism may be related to common genetic variations that are associated with NAFLD, such as the case of PNPLA3 Ile148Met (rs738409) isoforms, as observed in in vitro studies based on knocking down or over-expression of the polymorphism lIe148Met.

PNPLA3 seems to have a critical role in the modulation of liver metabolism beyond its classical participation in triacylglycerol remodeling [43]. Finally, combining NAFLD-histological variables, levels of circulating metabolites, and genetic markers in a two-stage multicenter case-control study, Sookoian et al. observed decreased levels of betaine in circulation in NASH and an association of genotypes of the missense variant p. Ser646Pro (rs1805074) in DMGDH gene, which encodes for the mitochondrial dimethyl glycine dehydrogenase with disease severity [44]. The available studies (Figure 2), reviewed also in Gitto et al. [45], showed that metabolomic patterns are different in patients with NAFLD, compared to healthy controls. However, the discrimination between NAFL and NASH remains a true challenge.

## 6. OMICS Data and System Biology Integration

Data derived from single-omics analysis are not enough to explain the complexity of liver diseases. Integration of multiomics data with biological network models will allow advances in our understanding of the complex biochemical processes and pathophysiological responses in liver diseases [46,47]. Moreover, it is also important to integrate gene products, mRNA, proteins, and metabolites, as well as their molecular interactions with the environmental factors (such as diet) [48,49]. Several attempts have been made in order to obtain information useful to characterize complex phenotypes in humans [50] by integrating Omics datasets using systems biology tools. As shown by Subramanian and colleagues [51], the application of gene set enrichment analysis (GSEA) to the genomic data sheds new light on the shared disease pathways between alcoholic and nonalcoholic liver disease. Same approaches have been utilized on metabolimics data. The metabolites set enrichment analysis (MSEA) compares the metabolic signature—metabolites that are overexpressed—with the whole set of metabolites found in known metabolic pathways. The MSEA has been applied by Dumas et colleagues [52] to show alterations in the metabolic pathways associated with NAFLD. Recently, Pirola et al. [5] performed an OMIC s integrative analysis, selecting a list of genes associated with NAFLD and metabolites known to be altered in NAFLD and NASH and observed interesting results on some pathways involved in NAFLD pathophysiology: the ATP binding cassette family (ABCC) and solute carriers transporters (SLC). These data need to be further explored.

## 7. Conclusions

OMICs-derived biomarkers in the management and treatment of patients with NAFLD are still under extensive evaluation. Their validation and replication are mandatory before they can be used as diagnostic markers to identify patients at risk of advanced disease, including liver cancer. In the future, integrating OMICs with clinical data will hopefully lead to a personalized NAFLD “molecular signature” useful for diagnosis as well as treatment, including “personalized drugs”, even though a healthy life style, diet, and exercise still remain the foundation for prevention and therapy.

## Figures and Tables

**Figure 1:** OMICs’ description and application.

**Figure 2:** OMICs signatures/biomarkers and NAFLD severity.
